# Antitumor Effect of Si-Jun-Zi Decoction on SGC7901 Gastric Cancer Cells by CMTM2 Activation

**DOI:** 10.1155/2022/4675815

**Published:** 2022-07-14

**Authors:** Xiangnan Li, Wenna Chen, Lanying Miao, Hongwei Sun, Xia Gao, Shengnan Guo, Yueshi Zhang, Yufeng Yang, Junfu Guo

**Affiliations:** ^1^Teaching and Experiment Center, Liaoning University of Traditional Chinese Medicine, Shenyang 110847, Liaoning, China; ^2^Department of Medical Laboratory Science, Liaoning University of Traditional Chinese Medicine, Shenyang 110847, Liaoning, China; ^3^Department of Laboratory, Second Affiliated Hospital of Dalian Medical University, Dalian 116027, Liaoning, China

## Abstract

The Si-Jun-Zi decoction (SJZ), a traditional Chinese medicine (TCM) formula, is used clinically against multiple malignancies, including gastric cancer (GC). In previous study, we have shown that SJZ plays an anticancer role in SGC7901 cell xenograft mice models. However, the underlying mechanisms are unclear. The objective of this study was to evaluate the effect and mechanism of SJZ on the proliferation, migration, invasion, and cancer stem cell-like properties of GC cells. High-throughput mRNA sequencing analysis was performed to investigate the global alterations in gene expression in xenograft tumors, and 56 significantly differentially expressed genes (43 upregulated and 13 downregulated genes) were identified between the SJZ group and the Model group totally. We focused on CMTM2, which was significantly increased after SJZ intervention, as a candidate target gene of SJZ. The results indicated that CMTM2 expression was elevated in SJZ-treated SGC7901 cells and knocking-down *CMTM2* expression partially hampered the inhibitory effects of SJZ on the proliferation, migration, and invasion of GC cells. Moreover, SJZ treatment repressed the spheroid and colony-forming capacity in GC cells, accompanied by downregulation of stem cell markers including SOX2, NANOG, and CD44. *CMTM2* knockdown antagonized the effects of SJZ on the cancer stem cell-like properties of SGC7901 cells. Thus, SJZ effectively suppressed the proliferation, migration, invasion, and cancer stem cell-like properties of GC cells *in vitro* by upregulating CMTM2 expression.

## 1. Introduction

Gastric cancer (GC) is the most common gastrointestinal tumors and the third leading cause of cancer death globally. [1, 2] Over the past decades, although 5-year survival rate of GC has rapidly increased thanks to significant improvements in diagnosis rate of early GC, standardization of radical surgery, and chemotherapy, the mortality of patients with advanced-stage GC remains unfavorable. [3] Tumor relapse and metastasis are still major problems for patients with advanced GC. Consequently, it is urgent to explore adjuvant therapy of GC and investigate their molecular mechanisms underlying inhibition of recurrence and metastasis in GC treatment.

Recently, an increasing number of studies have verified that traditional Chinese medicine (TCM), which is usually used as a novel drug therapy of cancer, might play an antitumor role in suppressing treatment-resistant cancer cell proliferation, metastasis, and cancer stem cells in several cancers. [4–6] Si-Jun-Zi Decoction (SJZ) is a well-known TCM formula with the function of replenishing qi and strengthening the spleen based on Chinese medicine theory and has been used in gastrointestinal disease, including GC. [7–9] Clinically, SJZ treatment could lower the metastatic recurrence rate and reduce 3-year and 5-year death rates in GC patients compared with the chemotherapy group. [10] It was reported that modified SJZ treatment could reduce postoperative stress and inflammatory response, and enhance the T cell-mediated humoral immune response of patients with gastrointestinal tumors. [11] Furthermore, previous studies demonstrated that SJZ effectively inhibited the growth of tumors in nude mice-bearing xenografts from the human GC cell line, SGC7901. [12] *In vitro*, SJZ inhibits the proliferation of side population cells in GC cell lines by inducing cell apoptosis. [13, 14]

Our previous studies demonstrated that SJZ can inhibit proliferation and promote apoptosis of human GC MGC803 cells *in vitro* and plays an anticancer role in SGC7901 cell xenograft node mouse model, at least partly via modulating microRNA and paired target genes. [15, 16] To investigate the effects and mechanisms of SJZ in GC systematically, we performed high-throughput sequencing and bioinformatics analysis in SGC7901 cell xenograft node mouse model in this study. Our results indicated that CMTM2 (encoding CKLF-like MARVEL transmembrane domain-containing member 2) expression was significantly upregulated by SJZ intervention. CMTM2 is an immune-related gene belonging to CMTM2 family and closely related to tumor progression, recurrence, and prognosis in lung cancer, hepatocellular cancer, and GC. [17–19] However, the role of CMTM2 in GC progression is not fully elucidated. In the present study, we found that SJZ treatment elevated CMTM2 mRNA and protein expression levels, and suppressed the proliferation, migration, invasion, and cancer stem cell-like properties of GC cells. Moreover, knockdown of CMTM2 abrogated the effect of SJZ in GC cells. We speculated that SJZ suppressed the proliferation, migration, invasion, and cancer stem cell-like properties of GC cells *in vitro* may be through the activation of CMTM2.

## 2. Materials and Methods

### 2.1. Ethics Statement

All experiments performed in this study was conducted in accordance with the ethical standards according to the Declaration of Helsinki and national and international guidelines, and was approved by Attitude of the Animal Core and Welfare Committee of Liaoning University of Traditional Chinese Medicine.

### 2.2. Nude Mouse Subcutaneous Xenograft Model

Twelve BALB/C nude male mice (age, 6–8 weeks; weight, 20 ± 2 g; Beijing Huafukang Biotechnology Co., Ltd., Beijing, China) were subcutaneously injected 200 *μ*l of SGC7901 cell suspension (1 × 10^7^/mL). When the mean tumor volume reached approximately 100–200 mm^3^, the tumor-bearing mice were randomized into two groups: SJZ group (13.2 g/kg/day SJZ decoction) and Model group (saline only). Six mice were included in each group. After 3-week treatment, mice were euthanized and tumors were immediately removed, rapidly frozen in liquid nitrogen, and stored at −80°C for subsequent analyses.

### 2.3. High-Throughput mRNA Sequencing Analysis

Three tumor tissue samples from each group were randomly selected for mRNA sequencing and analysis. Total RNA extraction, detection, and transcriptome sequencing were carried out by Shanghai Personal Biotechnology Co., Ltd. (Shanghai, China). Briefly, RNA concentration and purity were determined by Agilent 2100 Bioanalyzer (Agilent Technologies, Santa Clara, CA, USA). Oligo (dT)-conjugated magnetic beads were used to enrich mRNA from total RNA. Subsequently, the RNA was broken into fragments of about 300 bp in length by ion interruption. First strand of cDNA was synthesized using 6-base random primers and reverse transcriptase, and the second cDNA strand was synthesized with the first cDNA strand as template. After RNA extraction, purification, and library construction, the libraries were paired-end (PE) sequenced using next-generation sequencing based on the Illumina HiSeq platform.

### 2.4. Bioinformatics Analysis

First, the Raw Data were filtered, and Clean Data obtained after filtering were mapped to the reference genome. The expression of each gene was calculated according to the comparison results. On this basis, the expression difference analysis, enrichment analysis, and cluster analysis were further carried out. Differentially expressed genes are annotated by Ensembl, GO, KEGG, EC, eggNOG, UniProtAC, NCBI_GI, and other databases, and differentially expressed mRNAs were screened based on following criteria: |log 2 (fold change)|≥1 and *p* < 0.05.

### 2.5. Preparation of SJZ-Treated Rat Serum

The main herbs in the SJZ formula (Chinese patent ZL201110145109.0) are *Radix Ginseng* (Renshen), *Poria cocos* (Fuling), *Rhizoma Atractylodis Macrocephalae* (Baizhu), and *Radix Glycyrrhizae* (Gan Cao) in a ratio of 3 : 3:3 : 2. These herbs were obtained from the first affiliated Hospital of Liaoning University of traditional Chinese medicine according to their original proportions. The medicine was decocted three times and concentrated into a stock solution (2.06 g of crude drug/ml).

Twenty specific pathogen-free (SPF) male rats (age, 8–10 weeks; weight, 350 ± 50 g; Liaoning Changsheng Biotechnology Co., Ltd., Benxi, China) were randomly divided into a control group (*n* = 10) and an SJZ group (*n* = 10). The control group was treated with 1 ml/100 g daily of normal saline (NS), and the SJZ group was treated with 1 ml/100 g (0.69 g/100 g body weight) daily of SJZ, once every day for a week. On the seventh day, the mice were anesthetized with 1% pentobarbital sodium; then, blood was taken from the abdominal aorta. The blood was centrifuged at 2000 ×g for 15 min at 1.5 h after drug treatment, and separated serum was collected. Then, the serum was incubated in a water bath for 30 min at 56°C, sequentially passed through 0.22-*μ*m filters for sterilization, and stored at −80°C until further use.

### 2.6. Cell Culture and Treatment

The human GC cell line SGC7901 was obtained from the Be Na Culture Collection (BNCC, Shanghai, China). Cells were cultured in Dulbecco's modified Eagleʼs medium (DMEM; HyClone, Logan, USA) containing 10% fetal bovine serum (FBS; Biological Industries, Beit HaEmek, Israel) and 1% penicillin-streptomycin (HyClone) and were maintained in a 5% CO_2_ incubator at 37°C. Cell passage was performed when the cells reached 80% of confluence.

SGC7901 cells (5 × 105–1 × 106 cells/well) were seeded in 6-well plates and treated with SJZ (DMEM containing 10% SJZ group serum) or NS (DMEM containing 10% control group serum). Cells were harvested at 48 h after treatment for use in the subsequent experiments.

### 2.7. Quantitative Real-Time Reverse Transcription (qRT-PCR)

Samples were exposed to Trizol (FOREGENE, Chengdu, China) for total RNA extraction. After cDNA was produced from total RNA by reverse transcription, the qPCR was performed using the SYBR Green Mixture (Bimake, Houston, TX, USA) according to the manufacture's procedure. The primers used are shown in Table 1. The PCRs comprised denaturation at 95°C for 5 min, followed by 40 cycles of 95°C for 15 s and 60°C for 60 s. GAPDH (encoding glyceraldehyde-3-phosphate) was used as an internal control. The relative mRNA expression was calculated using the 2^−ΔΔCt^ method [Table 1 near here].

### 2.8. Western Blotting

Whole-cell extracts were prepared using protein lysis buffer (Invent Biotechnologies, Plymouth, MN, USA). A bicinchoninic acid (BCA) protein assay kit (Fudebio, Hangzhou, China) was used to determine the protein concentrations. Total proteins (30 *μ*g) were separated using 10% SDS-PAGE and electrotransferred to polyvinylidene fluoride membranes. The membranes were blocked in 5% nonfat milk for 1 h at room temperature and then probed with primary antibodies against CMTM2 (ABP53869, Abbkine, Wuhan, China, 1 : 1000), SRY-box transcription factor 2 (SOX2) (11064-1-AP, Proteintech, Rosemont, IL, USA, 1 : 600), NANOG (67255-1-Ig, Proteintech, 1 : 10000), CD44 (15675-1-AP, Proteintech, 1 : 5000), and GAPDH (60004-1-Ig, Proteintech, 1 : 1000) overnight at 4°C. Subsequently, the membranes were incubated with goat anti-rabbit antibodies diluted with 0.3‰ in TBST (FDR007, Fudebio, Guangzhou, China, 1 : 10000) or goat anti-mouse antibody diluted with 0.3‰ TBST for 1 h at room temperature. The membranes were then scanned using the Tanon 5200 automated image analysis system (Tanon Science and Technology Co., Ltd, Shanghai, China), and the ImageJ software (National Institutes of Health) was used to evaluate the band intensity.

### 2.9. Cell Transfection

Duplex small interfering RNA (siRNA) oligonucleotides specific for human CMTM2 were synthesized by GenePharma (Shanghai, China). The siRNA sequences were as follows: 5′-CCAUGAAUCUCCACUACUUTT-3′ and 5′-AAGUAGUGGAGAUUCAUGGTT-3′. SGC7901 cells (5 × 105–1 × 106 cells/well) were cultured in 6-well plates, and 20 nM of the CMTM2 siRNA (si-CMTM2) or control siRNA (si-NC) was introduced into the cells using the jetPRIME transfection reagent (Polyplus Transfection, Illkirch, France) in accordance with the manufacturer's recommendations. After 4-h transfection, cell culture medium was changed to SJZ or NS culture medium for 48 h, and then, cells were harvested for subsequent experiments.

### 2.10. Cell Proliferation Assay

To quantify proliferation, SGC7901 cells (5 × 104–1 × 105 cells/well) were incubation with SJZ, NS, or SJZ after transfection of si-*CMTM2* or si-NC and placed into a Cytation 3 Cell Imaging Multimode Reader (BioTek Instruments, Winooski, VT, USA) containing a temperature and CO_2_-controlled chamber. Images were acquired at 0 h, 12 h, 24 h, 48 h, and 72 h after drug treatment or transfection using a 10× objective and were quantified using the Gen 5 data analysis software (BioTek Instruments).

### 2.11. Cell Scratch Assay

SGC7901 cells (5 × 105–1 × 106 cells/well) were seeded in 6-well plates and cultured in DMEM complete culture medium at 37°C. Confluent monolayers were scratched using a sterile 200-*μ*l pipette tip and washed gently with phosphate-buffered saline (PBS) to remove floating cells. The cells were then incubated with SJZ, NS, or SJZ after transfection of si-*CMTM2* or si-NC, and placed into a Cytation3 Cell Imager. Images were acquired at 0 h, 12 h, 24 h, 48 h, and 72 h after scratching using a 10× objective, and the covered areas were quantified using the Gen 5 data analysis software.

### 2.12. Cell Invasion Assays

The transwell inserts (Corning Inc., Corning, NY, USA) were precoated with Matrigel (Corning Inc., Corning, NY, USA). Then, SGC7901 cells (1 × 10^4^ cells/well) were resuspended in DMEM culture medium containing 10% FBS after different treatments and seeded into the upper chambers of inserts. The medium containing 20% FBS was placed in the bottom chambers. After 24 h of incubation, noninvading cells on the upper side of the filter were gently removed with a cotton swab. Then, the insert was stained with 0.1% crystal violet for 20 min. Using an inverted microscope (Nikon, Tokyo, Japan), cells in five random fields were visualized and enumerated with the ImageJ software (National Institutes of Health). All experiments were performed in triplicate.

### 2.13. Cell Spheroid Formation Assay

SGC7901 cell suspensions (1 × 103 cells/well) were plated in 24-well ultra-low attachment plates (Corning Inc., Corning, NY, USA) after different treatments and maintained in serum-free DMEM/F-12 medium containing 10 mmol/l HEPES, 20 ng/ml epidermal growth factor, 20 ng/ml basic fibroblast growth factor, 0.4% bovine serum albumin, and B27 supplement (1 : 50 dilution; Invitrogen, Waltham, MA, USA) for 7 days. The number of spheroids (diameter ≥75 *μ*m) was then counted in three random fields under an inverted microscope (Nikon, Tokyo, Japan).

### 2.14. Soft Agar Colony Formation Assay

SGC7901 cell suspensions (3 × 103 cells/well) were plated into 6-well plates after different treatments and maintained in DMEM containing 10% FBS and 0.3% low melting-point agarose (Solarbio, Beijing, China) on a base layer of 0.5% low melting-point agarose. After 7 days of incubation at 37°C, the number of colonies ≥50 *μ*m was counted and photographed in three random fields. Each experiment was performed in triplicate.

### 2.15. Statistical Analysis

All data are shown as the mean ± standard error of mean (SEM) and were analyzed using the GraphPad Prism 8.0. (GraphPad Software, La Jolla, CA, USA). Comparisons between two groups were assessed using an independent sample *t-*test, and comparisons among multiple groups were conducted using one-way analysis of variance. *P* < 0.05 was defined as statistically significant for all tests.

## 3. Results

### 3.1. Gene Expression Profiling in Tumor Tissues after SJZ Treatment

We conducted high-throughput sequencing analysis in tumor tissues from SGC7901 cell xenograft mice model. The result identified 56 significantly differentially expressed mRNAs (|log_2_fold change| 1.0, *p* < 0.05), including 43 upregulated and 13 downregulated genes, between the SJZ group and the Model group totally (Figure 1).

### 3.2. GO and KEGG Pathway Enrichment Analyses

In order to explore the biological functions of all these differentially expressed genes, we mapped them to terms in the Gene Ontology (GO) database, searching for significantly enriched GO terms compared with the reference gene background. GO enrichment analysis results of differentially expressed genes were selected by GO categories of molecular function (MF), biological process (BP), and cellular component (CC). The most significantly enriched terms for these three categories are “phosphatidylcholine transporter activity,” “extracellular region part,” and “lung alveolus development” (Figure 2).

The enrichment degree of Kyoto Encyclopedia of Genes and Genomes (KEGG) was measured by enrichment factors (Rich factor), FDR value, and the number of genes enriched in this pathway. The top 20 KEGG pathways with the most significant enrichment, including ABC transporters pathway, cholesterol metabolism pathway, cell adhesion molecule (CAMs) pathway, fat digestion and absorption pathway, and others, are displayed in Figure 3 [Figure 3 near here].

### 3.3. Validation of  mRNA Expression by qRT-PCR

To validate the results of mRNA sequencing, we selected 2 upregulated (*PTPN22* and *CMTM2*) and 3 downregulated (*KLK14*, *EREG,* and *TMEM238*) mRNAs for further assessment by qRT-PCR. Compared with those in the Model group, the mRNA expression levels of *PTPN22* and *CMTM2* in the SJZ group were obviously upregulated, and the mRNA expression levels of *KLK14*, *EREG,* and *TMEM238* were significantly downregulated (*P* < 0.01 or *P* < 0.001, Figure 4(a)). Generally, the qRT-PCR results were consistent with mRNA sequencing data and the correlation coefficient (*R*^2^) was 0.9816 (Figure 4(b)). Among all detected mRNAs, CMTM2, an immune-related gene, had a 3.07-fold increase in expression after SJZ treatment by qRT-PCR analysis, similar to that detected by mRNA sequencing (increased 4.04-fold), and was screened as a potential candidate target of SJZ (Figure 4).

### 3.4. SJZ Upregulates the Expression of CMTM2 in GC Cell Lines

To further explore the biological function of CMTM2 in GC, we first verified CMTM2 expression in GC cell line SGC7901 after SJZ or NS treatment by qRT-PCR and western blotting. As shown in Figure 5(a) and 5(b), the expression of CMTM2 mRNA and protein was significantly higher after SJZ treatment than NS treatment (*P* < 0.01 or *P* < 0.001). These results showed that SJZ upregulated the expression of CMTM2 in GC cells (Figure 5).

### 3.5. SJZ Modulates GC Cell Proliferation via CMTM2

We determined transfection efficiency by qRT-PCR and western blot prior to cell function assays. The results showed that the expression level of CMTM2 in SJZ-treated SGC7901 cells with si-*CMTM2* transfection was significantly lower than si-NC transfection (*P* < 0.01, Figure 6(a) and 6(b)). The data indicated the high transfection efficiency of cells.

Cell proliferation assay was performed by live cell imaging and showed that the cell proliferation rate decreased significantly in the SJZ group compared with that in the NS group at 24 h, 48 h, and 72 h, while *CMTM2* knockdown accelerated the cell proliferation of SGC7901 cells significantly (*P* < 0.01 or *P* < 0.001, Figures 6(c) and 6(d)). The above findings indicated that SJZ repressed the proliferation of GC cells through upregulation of *CMTM2* expression *in vitro* (Figure 6).

### 3.6. SJZ Modulates GC Cell Migration and Invasion via CMTM2

To further evaluate the role of CMTM2 in the metastasis of SJZ-treated GC cells, cell scratch assay and invasion assay were conducted in SGC7901 cells. As shown in Figure 7, SJZ impeded the migrating and invasive capabilities of SGC7901 cells, while *CMTM2* knockdown antagonized the effect of SJZ (*P* < 0.05 or *P* < 0.001). These results showed that decreased CMTM2 expression could partially reverse the inhibition of cell migration and invasion induced by SJZ in GC cells [Figure 7 near here].

### 3.7. SJZ Modulates GC Cell Spheroid and Colony Formation via CMTM2

The spheroid assay demonstrated that SJZ treatment markedly reduced the number of spheroids (Figure 8(a) and 8(b), *P* < 0.01), whereas *CMTM2* knockdown yielded the opposite effects in SGC7901 cells (Figures 8(a) and 8(b), *P* < 0.01). Consistently, the results from soft agar colony assay indicated that the colony number decreased in the SJZ group compared with the NS group (Figures 8(c) and 8(d), *P* < 0.001), while the colony number increased after *CMTM2* knockdown (Figures 8(c) and 8(d), *P* < 0.01). These above results suggested that SJZ might regulate the cell spheroid and colony formation by modulating CMTM2 expression in GC cells (Figure 8).

### 3.8. SJZ Modulates the Expression of Stem Cell Markers SOX2, NANOG, and CD44 via CMTM2

To further investigate the relationship between cancer stem cell-like properties and CMTM2, we detected the expression of stem cell markers SOX2, NANOG, and CD44 in SGC7901 cells using qRT-PCR and western blotting. As shown in Figure 9(a), the expression levels of *SOX2*, *NANOG*, and *CD44* mRNA were reduced significantly by SJZ treatment in SGC7901 cells (*P* < 0.011). Furthermore, there was an increase in the expression of *SOX2*, *NANOG*, and *CD44* after *CMTM2* knockdown followed by SJZ treatment in SGC7901 cells (Figure 9(a), *P* < 0.05 or *P* < 0.01). Consistent with qRT-PCR results, a marked reduction in the protein levels of SOX2, NANOG, and CD44 was observed after SJZ treatment in SGC7901 cells, an effect that was rescued by *CMTM2* knockdown (Figure 9(b), *P* < 0.05, *P* < 0.011 or *P* < 0.001). Taken together, these data showed that SJZ repressed the expression of SOX2, NANOG, and CD44 via CMTM2 in GC cells (Figure 9).

## 4. Discussion

The classic recipe SJZ was first reported in a traditional pharmacopoeia named “Taiping Huimin Heji Jufang” in Song Dynasty of China, which is a representative recipe for improving gastrointestinal function and regulating human body's immune system. [20] However, the anticancer targets and pharmacological mechanisms of SJZ have not yet been clarified because of its complex composition. Our previous study demonstrated that SJZ altered miRNA expression profiles and inhibited expression of their target genes, thus affected biological functions of GC cells including proliferation, apoptosis, migration, and cancer stem cell-like properties. [16] Therefore, in the current study, we screened potential targets of SJZ by high-throughput mRNA sequencing and investigated the effects and mechanisms of SJZ on the proliferation, migration, invasion, and cancer stem cell-like properties of the GC cell line SGC7901.

First, 56 differentially expressed genes (43 upregulated and 13 downregulated) were identified and CMTM2 was significantly elevated after intervention of SJZ in xenograft mice model. Then, we verified that the expression of *CMTM2* mRNA was elevated by SJZ treatment in both tumor tissues and GC SGC7901 cells by qRT-PCR. It was reported that the expression of transcription factor *CMTM2* was remarkably lower in GC tissues than that in paired adjacent normal tissues, and was shown to participate in the inhibition of long noncoding RNA LINC01391 on cell migration, invasion, and aerobic glycolysis in GC SGC7901 cells. [21] Downregulated *CMTM2* promotes the metastasis of hepatocellular carcinoma via inducing the EMT process. [19] In addition, a study identified a significant novel mutation in CMTM2 in diffuse-type GC and overexpressed CMTM2 significantly suppressed GC cells proliferation. [22] Downregulation of AP-1 inhibits drug resistance in SGC7901 GC cells, while CMTM2 selectively inhibited AP-1 activity. [23, 24] These studies suggested a potential anticancer role of CMTM2 in tumor aggressiveness and drug resistance. Thus, CMTM2 might be a potential target of SJZ. Accordingly, the effect of CMTM2 on the proliferation, migration, and invasion of GC cells was investigated. We discovered that SJZ restrained the proliferation, migration, and invasion of GC cells. Meanwhile, knockdown of *CMTM2* in GC cells could partially reverse these effects of SJZ. Therefore, we provided evidence that CMTM2 mediated the inhibitory effect of SJZ on the development of GC cells.

Recent studies have proven that cancer stem cells are a rare population of cancer cells with the potential of self-renewal, multidirectional differentiation, infinite proliferation, and tumor reconstruction, and are associated with metastasis and resistance to chemotherapeutic drugs. [25, 26] It has been identified that cancer stem cells exist in various types of tumors, including those in the brain, [27] lung, [28] breast, [29] liver, [30, 31] pancreas, [31] prostate, [32] ovary, [33] melanoma, [34] mesenchymal carcinomas, [35] and gastrointestinal tumor. [36] In the case of GC, the existence of GC stem cells was firstly suggested by Takaishi et al. [37] Subsequent studies have recognized the existence and pathological significance of GC stem cells or the cancer stem cell-like characteristics of GC cell lines and GC tissues. [6, 38–40] Thus, GC stem cells have become an important target for therapeutic interventions in GC.

Ginsenoside F2, an active ingredient of famous Chinese traditional herbs Ginseng (the main herb of SJZ), induces cancer stem cell apoptosis and initiates autophagy through promoting endogenous apoptosis pathways and mitochondrial dysfunction. [41, 42] *KLF4* (encoding Kruppel-like factor 4), as a major cancer stemness-related gene, has been reported to be a potential therapeutic target of SJZ for the treatment of colorectal cancer. [43] These studies support the close relationship between SJZ and cancer stem cell-like properties. Therefore, we investigated the role of SJZ in the cancer stem cell-like properties of SGC7901 cells. The early transcription factors SOX2 and NANOG are regulatory factors of GC stem cells and maintain the ability of pluripotency, self-renewal, and differentiation in both embryonic and adult stem cells. [44–46] As a universal cancer stem cell marker, CD44 has been identified in sorts of cancer cell lines and primary tumors including GC. [47, 48] The CD44-positive expression percentage in GC cells was strongly associated with tumor recurrence and progression. [49] It was also reported that GC stem cells, isolated from the SGC7901 GC cell line, highly expressed stem cell surface markers, including SOX2, NANOG, and CD44. [50, 51] Thus, we selected SOX2, NANOG, and CD44 as GC stem cell markers. Our results showed that SJZ treatment inhibited the spheroid and colony-forming capacities of SGC7901 cells, accompanied by downregulation of cancer stem cell markers such as SOX2, NANOG, and CD44. In addition, knockdown of CMTM2 could antagonize the effects of SJZ on SGC7901 cells' expression of SOX2, NANOG, and CD44 and their cancer stem cell-like properties. These findings indicated a significantly inhibitory effect of SJZ on cancer stem cell-like properties of GC cells, which is associated with SJZ-induced CMTM2 upregulation. These findings further support the suppressive role of CMTM2 in GC cell pathogenesis and disease progression.

Immune-related genes are important targets for immunotherapy of cancer and widely applied in the clinical. [52] CMTM2 is one of immune-related genes and has a protective effect on some carcinomas. [18] *Helicobacter pylori* infection-related chronic inflammation is a leading cause of gastric cancer. [53] It has been reported that SJZ positively regulates innate immune response by increasing macrophages and is beneficial for gastrointestinal system. However, the influence of CMTM2 in SJZ regulation of immune response in GC needs to be further explored.

In conclusion, we examined differentially expressed mRNAs from high-throughput sequencing in SGC7901 xenograft tumor model, followed by experimental validation to investigate target gene involved in the antigastric cancer effects of SJZ in SGC7901 GC cell line. We verified SJZ upregulated CMTM2 expression in GC cell line in both gene transcription level and protein level by qRT-PCR and western blot. Then, the inhibitory effects of SJZ on the proliferation, migration, invasion, and cancer stem cell-like properties of GC cells were detected by live cell imaging, cell invasion assays, cell spheroid formation assay, and soft agar colony formation assay. Furthermore, we found that the biological effects of GC cells produced by SJZ treatment partially depend on CMTM2 upregulation by transfection with si-CMTM2. Our research illustrated an important function of SJZ in the malignant behaviors of GC, and its mechanism might be related to CMTM2 and its target pathways.

## Figures and Tables

**Figure 1:** Volcano plot analysis of the differentially expressed mRNAs in the SJZ group compared with the Model group. The expression of 56 genes was significantly changed (>1-fold, *P* < 0.05). A total of 43 genes were upregulated, and 13 genes were downregulated. *x*-axis parallel lines, *P* value = 0.05. *y*-axis parallel lines, log_2_ (fold change)  = 1. Red areas indicate an upregulated mRNA, blue indicates a downregulated mRNA, and grey indicates no significant changes in mRNA expression.

**Figure 2:** GO analysis of the differentially expressed mRNAs in the SJZ group relative to the Model group (top 10 enriched terms of cellular components, molecular functions, and biological processes were displayed).

**Figure 3:** KEGG analysis of the differentially expressed mRNAs in the SJZ group relative to the Model group (top 20 enriched pathways).

**Figure 4:** The qRT-PCR-based validation of differentially expressed genes. (a) The relative expression levels of *PTPN22*, *CMTM2*, *KLK14*, *EREG,* and *TMEM238* mRNA in tumor tissue and (b) correlation analysis of log_2_ (fold change) values measured using qRT-PCR and mRNA sequencing methods. ^*∗∗*^*P* < 0.01 and ^*∗∗∗*^*P* < 0.001, compared with the Model group.

**Figure 5:** SJZ upregulates the expression of CMTM2 in GC cells. The expression of (a) CMTM2 mRNA and (b) protein in SGC7901 GC cells after incubation with SJZ or NS for 48 h was detected using qRT-PCR and western blotting, respectively. ^*∗∗*^*P* < 0.01 and ^*∗∗∗*^*P* < 0.001 compared with the NS group.

**Figure 6:** SJZ modulates cell proliferation via CMTM2. (a) The mRNA and (b) protein expression of CMTM2 in SJZ-treated SGC7901 cells after transfection of *CMTM2* siRNAs (SJZ + si-*CMTM2*) or negative control siRNAs (SJZ + si-NC), as detected using qRT-PCR and western blotting, respectively. NC, negative control; si-*CMTM2* are siRNAs targeting *CMTM*2. (c) Representative images of cell proliferation assay of SGC7901 cells after incubation with SJZ, NS, or SJZ after transfection of si-*CMTM2* or si-NC at 0-h and 72-h magnification, ×100. (d) Cell proliferation rate of SGC7901 cells after treatment. ^*∗∗*^*P* < 0.01 and ^*∗∗∗*^*P* < 0.001 compared with the control.

**Figure 7:** SJZ modulates cell migration and invasion via CMTM2. (a) Representative images of cell scratch assay of SGC7901 cells treated with SJZ, NS, or SJZ after transfection of si-*CMTM2* or si-NC at 0-h, 24-h, and 48-h magnification, ×100. (b) Relative covered area of SGC7901 cells after treatment. (c) Representative images of cell invasion assay of SGC7901 cells after treatment; magnification, ×100. (d) The mean number of invaded cells from five randomly selected fields under the microscope. ^*∗*^*P* < 0.05 and ^*∗∗∗*^*P* < 0.001 compared with the control.

**Figure 8:** SJZ modulates cell spheroid and colony formation via CMTM2. (a) Representative images of spheroids formed by SGC7901 cells treated with SJZ, NS, or SJZ after transfection of si-*CMTM2* or si-NC; magnification, ×100. (b) The mean number of spheroids calculated in three randomly selected fields under the microscope. (c) Representative images of colonies formed by SGC7901 cells after treatment; magnification, ×100. (d) The mean number of colonies calculated in three randomly selected fields under the microscope. ^*∗∗*^*P* < 0.01 and ^*∗∗∗*^*P* < 0.001 compared with the control.

**Figure 9:** SJZ modulates the expression of stem cell markers SOX2, NANOG, and CD44 via CMTM2. (a) The expression levels of SOX2, NANOG, and CD44 mRNA and (b) protein in SGC7901 cells incubation with SJZ, NS, or SJZ after transfection of si-CMTM2 or si-NC were detected using qRT-PCR and western blotting, respectively. ^*∗*^*P* < 0.05, ^*∗∗*^*P* < 0.01, and ^*∗∗∗*^*P* < 0.001 compared with the control.

**Table 1:** Primer sequences of for the genes investigated in the present study.

Genes	Sequence
*CMTM2*	F: 5′-TTTCTGACCTCTTCAACGACCT-3′
	R: 5′-AAACTCCAGCCGCACCAATA-3′
*PTPN22*	F: 5′-CCAGCTACATCAATGCCAACTTC-3′
	R: 5′-CCAAATCATCCTCCAGAAGTCC-3′
*KLK14*	F: 5′-CAGCCCCTAAAATGTTCCTCC-3′
	R: 5′-TGCACGTATGGCCACCAAT-3′
*EREG*	F: 5′-ATCCTGGCATGTGCTAGGGT-3′
	R: 5′-GTGCTCCAGAGGTCAGCCAT-3′
*TMEM238*	F: 5′-CTTCGGGGACCTGCTCATCT-3′
	R: 5′-GGGTTGTCTGGGCCTCACTC-3′
*SOX2*	F: 5′-GAAAAACGAGGGAAATGGG -3′
	R: 5′-GCTGTCATTTGCTGTGGGT-3′
*NANOG*	F: 5′-CCTCCTCCCATCCCTCATA-3′
	R: 5′-TGATTAGGCTCCAACCATACTC-3′
*CD44*	F: 5′-CATCCCAGACGAAGACAGTCC-3′
	R: 5′-TGATCAGCCATTCTGGAATTTG-3′
*GAPDH*	F: 5′-ATCATCAGCAATGCCTCC-3′
	R: 5′-CATCACGCCACAGTTTCC-3′

## Data Availability

The datasets used and analyzed during the current study are available from the corresponding author upon reasonable request.
